# Face Mask-Wearing Detection Model Based on Loss Function and Attention Mechanism

**DOI:** 10.1155/2022/2452291

**Published:** 2022-07-12

**Authors:** Zhong Wang, Wu Sun, Qiang Zhu, Peibei Shi

**Affiliations:** School of Computer Science and Technology, Hefei Normal University, Hefei 230601, China

## Abstract

Face mask-wearing detection is of great significance for safety protection during the epidemic. Aiming at the problem of low detection accuracy due to the problems of occlusion, complex illumination, and density in mask-wearing detection, this paper proposes a neural network model based on the loss function and attention mechanism for mask-wearing detection in complex environments. Based on YOLOv5s, we first introduce an attention mechanism in the feature fusion process to improve feature utilization, study the effect of different attention mechanisms (CBAM, SE, and CA) on improving deep network models, and then explore the influence of different bounding box loss functions (GIoU, CIoU, and DIoU) on mask-wearing recognition. CIoU is used as the frame regression loss function to improve the positioning accuracy. By collecting 7,958 mask-wearing images and a large number of images of people without masks as a dataset and using YOLOv5s as the benchmark model, the mAP of the model proposed in the paper reached 90.96% on the validation set, which is significantly better than the traditional deep learning method. Mask-wearing detection is carried out in a real environment, and the experimental results of the proposed method can meet the daily detection requirements.

## 1. Introduction

The spread of COVID-19 endangers public safety, and its known transmission routes mainly include droplet transmission and close contact. Therefore, wearing masks has become the main means of preventing the spread of the virus [1, 2]. The traditional methods of inspecting mask-wearing are mostly manual inspections, which not only consume manpower and material resources and are inefficient but also cause certain difficulties in personnel management, which is more likely to cause crowds to gather and increase the risk of virus spread.

Mask-wearing detection technology is one of the key prevention means supervised by epidemic prevention departments, and the stability and robustness of mask detection algorithms are particularly important. Mask-wearing detection is developed based on face detection and target classification. Compared with simple face detection, mask-wearing detection needs to address many problems, such as different lighting, side faces, occlusion, and density. However, solving these problems and improving mask-wearing detection accuracy are of great significance [3, 4].

With the development of deep learning technology, mask-wearing detection technology based on deep learning has been widely used [5, 6]. However, due to the influence of a complex environment, the existing algorithms have the problems of low accuracy and slow detection speed, which cannot achieve real-time detection. To this end, based on the YOLOv5 model, this paper introduces an attention mechanism to selectively enhance the fused features, highlight important features, reduce the impact of redundant features, and use the CIoU loss function as a new bounding regression loss function to make the regression of the target model more documented and the positioning more accurate. The main contributions of the paper are as follows:

1. Study the effect of different attention mechanisms (CBAM, SE, and CA) on improving the deep network model.
2. Explore the impact of different bounding box loss functions (GIoU, CIoU, and DIoU) on mask-wearing recognition.

The rest of the content is arranged as follows: Section 2 introduces the work related to mask-wearing detection.  Section 3 focuses on describing the framework and implementation details of the mask-wearing detection model.  Section 4 verifies the performance of the proposed method through experimental tests and finally gives a summary and outlook.

## 2. Related Works

Mask-wearing detection is an object detection task that determines the location and category of each object in the image. Mask-wearing detection methods based on deep learning are divided into two categories. One is a two-stage target detection model based on region extraction, such as RCNN (regions convolutional neural networks) [7], Fast R-CNN [8], Faster R- CNN [9], R-FCN [10], Cascade R-CNN [11], and DeRPN [12], which divide the target detection into two steps: feature extraction and feature classification. The other is to obtain the classification results directly based on the regression method, which can realize real-time detection in terms of detection speed, but it is slightly insufficient in detection accuracy, such as SSD (single shot multibox detector) [13], YOLO (you only look once) [14, 15] series, RetinaNet [16], and RefineDet [17]. Recently, researchers have proposed various mask-wearing detection technologies based on the above methods. Fan and Jiang [18] proposed a high-performance single-stage mask-wearing detector named RetinaFaceMask, which includes a new dataset, a contextual attention module, and transfer learning. Jignesh Chowdary et al. [19] proposed a transfer learning model to automatically detect mask-wearing, which was performed by fine-tuning the pretrained InceptionV3 model. Rahman et al. [20] proposed a system to limit the growth of COVID-19 by using deep learning models and cameras to discover people who are not wearing masks in urban networks. Loey et al. [21] proposed a hybrid model based on deep learning and classical machine learning, including two parts: the first part uses ResNet50 for feature extraction, and the second part uses SVM and ensemble algorithms for classification. Ren and Liu [22] designed a YOLOv3-based convolutional neural network named Face_mask Net.

Attention mechanisms have achieved great success in various computer vision tasks [23]. The purpose of introducing an attention mechanism is to select key information from many redundant pieces of information to submit the detection ability of the network. Attention-based models include four stages in the field of computer vision: combining deep neural networks with attention mechanisms, representative methods include RAM [24]; in explicit prediction of discriminative input features, representative methods include STN [24, 25] and DCN [26]; to implicitly and adaptively predict potential key features, representative methods are SENet [27], CBAM [28], and CA [29]; attention methods are related to the self-attention mechanism, and the representative methods are nonlocal [30] and ViT [31]. Attention mechanisms are also divided into channel attention, spatial attention, temporal attention, branch attention, and multiple class mixing methods.

Bounding box regression is a mainstream technique in object detection that uses a rectangular bounding box to predict the location of the target object in the image, aiming to refine the predicted bounding box location. Bounding box regression adopts the overlapping area between the predicted bounding box and the ground-truth bounding box as the loss function, which is called the IoU-based loss function. Deep learning optimization suffers when the predicted and ground-truth bounding boxes do not intersect. GIoU [32] is an improvement on IoU. While maintaining the advantages of IoU, it also addresses other non-overlapping regions, reflecting the degree of overlap between the two to a certain extent. DIoU [33] considers the overlapping area and the center point distance. When the target frame wraps the prediction frame, it directly measures the distance between the two frames, so the convergence is faster. Based on DIoU, CIoU uses the aspect ratio of the prediction box and the target box as an impact factor. Alpha-IoU [34] can significantly outperform existing IoU-based losses and is more robust to small datasets and noise. Aiming at the problem of dense targets in mask recognition, Zhang et al. [35] proposed to learn the IoU-Aware classification score and design a new loss function named Varfocal Loss to propose a new bounding box feature representation method for prediction and boundary refinement. At the same time, real-time mask-wearing detection [36, 37] and transfer learning methods [38–40] have been widely studied. For example, Mahmoud et al. [36] proposed a real-time feature extraction module based on deep convolutional neural network. Xu [37] proposed a lightweight YOLOv5 model and used alpha-CIoU as the loss function. Mercaldo and Santone [38] proposed a transfer learning method that uses the MobileNetV2 model to identify illegal mask-wearing behaviors in videos. Su et al. [39] proposed a mask-wearing recognition method that integrates transfer learning and Efcient-Yolov3, using EfcientNet as the backbone network and CIoU as the loss function.

## 3. Methodology

### 3.1. Improved YOLOv5

YOLOv5 is a representative of a single-stage detection model, which has the advantages of fast speed and high accuracy. Compared with YOLOv4, the model has fewer parameters, simple operation, and easier transplantation to the mobile terminal. It was proposed by Ultralytics in May, 2020. There are four network models, namely, YOLOv5s, YOLOv5m, YOLOv5l, and YOLOv5x. Among them, YOLOv5s has the smallest network depth and feature map width, and the other three models are continuously deepened and widened based on YOLOv5s.

Based on YOLOv5s, this paper adds the CBAM attention mechanism in the feature fusion process to improve feature utilization and uses CIoU as the bounding loss function to improve the positioning accuracy. The model structure is shown in Figure 1. The improved model is the same as the traditional YOLOv5s, including four parts: input, backbone, neck, and prediction:

1. The input includes an adaptive anchor box and an adaptive image scaling.
2. The backbone includes the focus module and the CSP module. The slicing operation in the focus module reduces the number of computations and improves the speed while realizing downsampling. The CSP module is beneficial for improving the network learning ability and reducing the memory cost. Two structures, CSP1 and CSP2, are designed in YOLOv5s. The CSP1 structure and the CSP2 structure are applied to the backbone and neck networks, respectively, to further speed up the inference speed of the network model.
3. The core of the neck adopts FPN and PAN structures. The FPN and PAN structures realize the fusion and complementation of high-level features and low-level features. FPN is top-down and uses upsampling process to transfer and fuse the new type to obtain the predicted feature map. The PAN adopts a bottom-up feature pyramid. In this paper, CBAM is introduced into FPN, and the fused feature map is sent to CBAM to reduce the influence of redundant features after fusion.
4. The prediction includes the bounding box loss function and nonmaximum suppression (NMS). In this paper, CIoU is used as the loss function to locate the target box more accurately. In the target detection prediction result processing stage, the optimal target frame is obtained by using the weighted NMS operation for screening numerous target frames.

### 3.2. Attention Mechanism

The convolutional block attention module (CBAM) is a lightweight convolutional attention module that combines channel and spatial attention mechanism modules. CBAM includes two submodules, the channel attention module (CAM) and the partial attention module (SAM), which perform channel and spatial attention, respectively. This not only saves parameters and computing power but also ensures that it can be integrated into the existing network architecture as a plug-and-play module. CAM is an adjustment to the structure of the SE module. Based on the SE module, a global maximum pooling operation is added to the CAM. CAM compresses the feature map into a one-dimensional vector in the spatial dimension, uses global average pooling and global maximum pooling to aggregate the feature information of the spatial map, and performs an element-by-element sum operation on the results by sharing the fully connected layer. The structure setting of the double pooling operation can make the extracted high-level features richer and provide more detailed information. SAM performs the concatenating operation on the result of the CAM operation based on the channel and performs single-channel dimensionality reduction through convolution. Similar to CAM, SAM adopts a double pooling operation. CBAM is similar to the SE module. The module structure mostly uses a 1 × 1 convolution to operate and completes the information extraction of the feature map through the entire channel dimension of the SAM, as shown in Figure 2.

Since the CBAM model adds a global maximum pooling operation to the CAM, it can make up for the information lost by the global average pooling to a certain extent. In addition, the generated 2D spatial attention map is encoded using a convolutional layer with a kernel size of 7, and a larger kernel is good for preserving important spatial regions. The YOLOv5s network with CBAM added can not only classify and identify the target more accurately but also locate the target more accurately.

### 3.3. Complete-IoU

The loss function of the target detection task consists of two parts: classification loss and bounding box regression loss. The most commonly used bounding box regression loss is IoU and its improved algorithm. The full name of the IoU algorithm is the intersection and union ratio, which is obtained by calculating the ratio of the intersection and union of the predicted box and ground-truth box, that is, IoU(*A*, *B*)=(*A*∩*B*)/(*A*∩*B*), where *A* is the predicted box and *B* is the ground-truth box. IoU can be used as the distance; then, Loss_IoU_=1 − IoU. The advantage of IoU is that it can reflect the detection effect between the predicted box and the ground-truth box. IoU has two disadvantages: when the prediction bounding box and the ground-truth bounding box do not intersect and IoU(*A*,*B*) = 0, the distance between *A* and *B* cannot be reflected. At this time, the loss function is not steerable and IoU loss cannot optimize the situation where the two bounding boxes do not intersect. Assuming that the sizes of the prediction bounding box and the ground-truth bounding box are determined, as long as the intersection value of the two boxes is determined and their IoU values are the same, the IoU value cannot reflect how the two boxes intersect. To this end, the paper adopts the CIoU loss function, and its formula is as follows:

(1) $$\begin{array}{c} \text{IoU}=\text{IoU}-\left(\frac{p^{2}\left(b,b^{gt}\right)}{c^{2}}+\alpha v\right),\\ \text{Loss}=1-\text{IoU}+\left(\frac{p^{2}\left(b,b^{gt}\right)}{c^{2}}+\alpha v\right),\\ v=\frac{4}{\pi^{2}}\left(\arctan\frac{w^{gt}}{\pi^{gt}}-\arctan\;{\frac{w}{h}}^{2}\right),\\ \alpha =\frac{v}{\left(1-\text{IoU}\right)+v}, \end{array}$$

where *b* and *b*^*gt*^ represent the center points of prediction box *B* and ground-truth box *B*^*gt*^, respectively, *c* represents the square of the diagonal length of the minimum bounding box *C*, *p* represents the calculation of the Euclidean distance between the two center points, *α* is the weight parameter, and *v* is used to measure the similarity of the aspect ratio. In addition, it can be seen that the CIoU loss function not only considers the overlapping area of the predicted frame and the real frame but also considers the distance between the center points and the aspect ratio of the two. Therefore, in the mask-wearing detection environment, the performance is better than other loss functions.

## 4. Experimental Results

### 4.1. Experimental Data and Environment

The paper collects 7,958 pictures of people wearing masks and not wearing masks in the network and real scenes as a dataset, including 7,158 training sets and 800 test sets. The ratio of the training set and test set is 9 : 1, and 0 and 1 are used to label the two categories. The sample images are shown in Figure 3.

The experimental environment of this paper was completed on the Ubuntu18.04 operating system. The GPU model is an NVIDIA GeForce RTX3060 12G, and the software environment is CUDA11 and PyTorch 1.7.

### 4.2. Evaluation Standard

In this paper, the precision rate, recall rate, average precision (AP), and mean average precision (mAP@0.5) are used as model accuracy evaluation indicators, where AP represents the area under the PR curve and mAP@0.5 represents the average precision (AP) of all categories when IoU is set to 0.5. The specific formula is as follows:

(2) $$\begin{array}{c} \text{precision}=\frac{\text{TP}}{\left(\text{TP}+\text{FP}\right)},\\ \text{recall}=\frac{\text{TP}}{\left(\text{TP}+\text{FN}\right)},\\ \text{AP}=\int_{0}^{1}P\text{d}R,\\ \text{mAP}=\frac{\sum_{i=1}^{N}AP_{i}}{N}, \end{array}$$

where TP is the number of correctly classified bounding boxes that are predicted and the bounding box coordinates that are correct, FN is the number of all unpredicted bounding boxes, and FP is the number of predicted bounding boxes that are misclassified or whose bounding box coordinates that are not up to the standard.

### 4.3. Experimental Results

In the training phase of the YOLOv5s model, the initial parameter batchSize is set to 8 and 8 images are randomly selected for training each time. The epoch is set to 450 rounds, and the rect is true. By setting the same parameters, different loss functions are used to train the network. When the model is trained to 300 epochs, the model begins to converge. After 450 epochs, each model takes the optimal result.

#### 4.3.1. Comparison of Attention Mechanisms

To verify the performance of the CBAM, this paper uses SE, CBAM, and CA to conduct comparative experiments. Among them, SE attention is channel attention, to solve the loss problem caused by the different weights occupied by different channels of the feature map in the process of neural network feature extraction. CBAM attention is additional spatial attention based on SE attention. The feature of CA is that the channel attention is divided into two different directions, horizontal and vertical, so that the information of the position and spatial direction of the input feature image can be fused, which can make the model more accurately locate the detection target.

By adding three attention mechanisms of SE, CBAM, and CA to different positions of the YOLOv5 network model (such as backbone network and neck network), the paper found that the performance of the same attention in different positions is different.  Table 1 presents the optimal results of different attention mechanisms, where CA is the worst and CBAM performs the best, which can improve mAP by 0.52% compared to the normal model without increasing the network complexity.  Figure 4 shows the comparison experiment curves based on the CBAM and the traditional network. It can be seen in the figure that adding the CBAM has a certain improvement effect.

#### 4.3.2. Comparison of Loss Functions

To verify the detection performance of the CIoU loss function, the paper uses IoU, GIoU, DIoU, alpha-IoU [34], and Varifocal [35] for comparative experiments. Among them, alpha-IoU (aIoU for short) is a unified exponentiation of existing losses based on IoU for accurate bbox regression and object detection. In this paper, the alpha-IoU is improved based on CIoU and the alpha is set to 2 and 3 for experimental comparison. When alpha = 1, it corresponds to the original CIoU loss function. Varifocal is a new loss function for training dense object detectors.

Table 2 presents the detection results of different loss functions. As can be seen from Table 2, CIoU is better than DIoU, GIoU, and aIoU and slightly lower than Varifocal.  Figure 5 represents the precision, recall, and mAP curves for different algorithms. When alpha = 3, the recall curve of aIoU-3 has obvious advantages. In addition, Figure 6 shows the detection result pictures based on Varifocal and CIoU. Although Varifocal achieves slightly better mAP, there will be obvious false positives in the case of the side face. Overall, the CIoU loss function is better.

To further verify the effectiveness of the method proposed in the paper, Table 3 also gives the traditional two-stage algorithm Faster R-CNN and the one-stage algorithm YOLOv3 as comparative experiments and uses mAP, precision, and recall to evaluate and compare each mainstream algorithm. Table 3 shows that the comprehensive performance of the network model proposed in the paper is the best; its mAP is 1.18% higher than that of Faster R-CNN and 4.85% higher than that of the YOLOv3 network model structure. After adding the CBAM to the backbone network, the performance of the network model is further improved and the final mAP reaches 90.96%.

Pictures of people wearing masks and pictures of people without masks in real scenes are collected, and the YOLOv5s + CIoU and YOLOv5s + CIoU + CBAM network models are used to evaluate the collected pictures. The detection results in the real environment are shown in Figure 7. As can be seen from the figure, the two face targets on the left are occluded. The above picture does not use the CBAM attention mechanism, resulting in missed detection, while the following picture can be applied to face detection under occlusion. From the above experimental results, YOLOv5s has occlusion and missed detection in the real environment. In contrast, the model proposed in this paper performs relatively well, especially for small target detection, which can achieve relatively accurate detection, but there is still missing detection in the shadow area. With the addition of the CBAM, the performance of the network model can be enhanced, corresponding with the expected experimental results.

## 5. Conclusion

Aiming at the occlusion and density problems of mask-wearing detection, this paper proposes a mask-wearing detection model based on an attention mechanism and loss function and carries out experimental tests based on different attention mechanisms and loss functions. Taking YOLOv5s as the basic framework, the experimental results show that the CBAM is significantly better than the other two attention mechanisms. Experimental tests on different loss functions show that the CIoU loss function is slightly better than the other three loss functions. The experimental results tested in the real environment show that the proposed model is robust to small targets and occlusion. Future work will further study the new network model to improve the accuracy of mask detection.

## Figures and Tables

**Figure 1:** The proposed model network structure.

**Figure 2:** Convolutional block attention module.

**Figure 3:** Sample images from the dataset.

**Figure 4:** Performance detection curves of different attention mechanisms.

**Figure 5:** Performance curves of different loss functions. (a) Precision. (b) Recall. (c) mAP@0.5.

**Figure 6:** Detection results with different loss function. (a) Varifocal. (b) CIoU.

**Figure 7:** Detection results with the proposed model. (a) YOLOv5s + CIoU and (b) YOLOv5s + CBAM + CIoU.

**Table 1:** The performance of different attention mechanisms.

Model	Precision (%)	Recall (%)	mAP@0.5 (%)
YOLOv5s + SE	95.00	84.03	89.70
YOLOv5s + CBAM	94.78	85.56	90.95
YOLOv5s + CA	95.15	76.91	82.51

**Table 2:** The performance of different loss functions.

Loss function	Precision (%)	Recall (%)	mAP@0.5 (%)
IoU	93.99	84.15	89.68
GIoU	93.87	85.24	90.17
DIoU	94.57	83.51	90.21
aIoU-2	95.13	85.06	89.87
aIoU-3	95.05	90.78	89.01
Varifocal	96.20	86.23	90.78
CIoU	93.69	84.90	90.43

**Table 3:** The performance of different models.

Model	Precision (%)	Recall (%)	mAP@0.5 (%)
YOLOv3	95.73	78.01	86.11
Faster R-CNN	72.99	90.51	89.78
YOLOv5s + CIoU	93.69	84.90	90.43
YOLOv5s + CBAM + CIoU	94.68	85.63	90.96

## Data Availability

The data used to support the findings of this study are included within the article.
